# Study of T2 mapping in quantifying and discriminating uterine lesions under different magnetic field strengths: 1.5 T vs. 3.0 T

**DOI:** 10.1186/s12880-022-00960-w

**Published:** 2023-01-04

**Authors:** Liuhong Zhu, Weihong Lu, Funan Wang, Yanwei Wang, Pu-Yeh Wu, Jianjun Zhou, Hao Liu

**Affiliations:** 1 Department of Radiology, Zhongshan Hospital (Xiamen), Fudan University, Jihun Road No. 668, Huli District, Xiamen, Fujian China; 2 Xiamen Municipal Clinical Research Center, Xiamen for Medical Imaging, Xiamen, 361015 China; 3 Department of Gynaecology Department, Zhongshan Hospital (Xiamen), Fudan University, Xiamen, Fujian China; 4 Department of Radiology, The Second Affiliated Hospital of Xiamen Medical College, Xiamen, Fujian China; 5 GE Healthcare, Beijing, China; 6 Department of Radiology, Zhongshan Hospital Fudan University, Xuhui District, Fenglin Road No.180, Shanghai, 200032 China

**Keywords:** T2 mapping, Transverse relaxation time, Adenomyosis, Endometrial cancer, Cervical cancer

## Abstract

**Background:**

MRI is the best imaging tool for the evaluation of uterine tumors, but conventional MRI diagnosis results rely on radiologists and contrast agents (if needed). As a new objective, reproducible and contrast-agent free quantification technique, T2 mapping has been applied to a number of diseases, but studies on the evaluation of uterine lesions and the influence of magnetic field strength are few. Therefore, the aim of this study was to systematically investigate and compare the performance of T2 mapping as a nonenhanced imaging tool in discriminating common uterine lesions between 1.5 T and 3.0 T MRI systems.

**Methods:**

A total of 50 healthy subjects and 126 patients with suspected uterine lesions were enrolled in our study, and routine uterine MRI sequences with additional T2 mapping sequences were performed. T2 maps were calculated by monoexponential fitting using a custom code in MATLAB. T2 values of normal uterine structures in the healthy group and lesions (benign: adenomyosis, myoma, endometrial polyps; malignant: cervical cancer, endometrial carcinoma) in the patient group were collected. The differences in T2 values between 1.5 T MRI and 3.0 T MRI in any normal structure or lesion were compared. The comparison of T2 values between benign and malignant lesions was also performed under each magnetic field strength, and the diagnostic efficacies of the T2 value obtained through receiver operating characteristic (ROC) analysis were compared between 1.5 T and 3.0 T.

**Results:**

The mean T2 value of any normal uterine structure or uterine lesion under 3.0 T MRI was significantly lower than that under 1.5 T MRI (*p* < 0.05). There were significant differences in T2 values between each lesion subgroup under both 1.5 T and 3.0 T MRI. Moreover, the T2 values of benign lesions (71.1 ± 22.0 ms at 1.5 T and 63.4 ± 19.1 ms at 3.0 T) were also significantly lower than those of malignant lesions (101.1 ± 4.5 ms at 1.5 T and 93.5 ± 5.1 ms at 3.0 T) under both field strengths. In the aspect of differentiating benign from malignant lesions, the area under the curve of the T2 value under 3.0 T (0.94) was significantly higher than that under 1.5 T MRI (0.90) (*p* = 0.02).

**Conclusion:**

T2 mapping can be a potential tool for quantifying common uterine lesions, and it has better performance in distinguishing benign from malignant lesions under 3.0 T MRI.

## Background

According to cancer statistics, the trend in the incidence and modality of uterine tumors in developing countries is still upward [1, 2]. Among uterine lesions, myoma and adenomyosis are the most common benign lesions, while cervical cancer and endometrial cancer are the most common malignant lesions, all of which threaten the health or life of patients. Currently, diagnostic curettage has become a widely used tool to screen uterine lesions. However, due to its invasive nature, there is a risk of complications such as pelvic inflammation caused by bacterial infection, amenorrhea caused by intrauterine adhesion, or even infertility. Among the noninvasive approaches, ultrasound is still the first choice for the diagnosis of uterine lesions due to its low cost and convenience. However, the low resolution and dependence on doctor experience limit its application in uterine lesion diagnosis and evaluation [3].

Magnetic resonance imaging (MRI) has become increasingly important in the diagnosis and evaluation of uterine lesions due to its non-radiation exposure and excellent image contrast of soft tissue. Lesion manifestations, such as shape, location, and signal intensity, on different contrast-weighted (such as T1- or T2-weighted) MRI images are the basis for radiologists to diagnose. The final diagnostic decision is radiologist dependent and subjective to a certain extent [4]. With the rapid development of MRI acquisition and reconstruction techniques and the big data era, the diagnosis of lesions is no longer limited to manifestations of contrast-weighted images and can benefit from quantitative measurements. As a quantitative technique, T2 mapping is objective, reproducible, stable, and suitable for patients with renal function insufficiency or gadolinium allergy due to its gadolinium-free nature [5]. It has been applied to a number of diseases, including prostate tumors [6, 7], breast tumors [8], ovarian cancer [9], uterine endometrial carcinoma [10], osteoarthritis [11, 12] and myocardial-related diseases [13, 14]. However, it is well known that the T2 value of certain tissues decreases with increasing magnetic field strength. Therefore, the influence of magnetic field strength, especially including the most commonly used 1.5 T and 3.0 T MRIs, should be taken into account during comparisons among different studies.

Therefore, our study aimed to systematically explore the feasibility of T2 mapping in quantifying common uterine lesions and to compare the performance of T2 mapping in discriminating common uterine lesions between 1.5 T and 3.0 T MRI systems.

## Materials and methods

### The principle of T2 mapping

There are various approaches for T2 mapping, such as multi-echo spin-echo (MESE) method [15], driven equilibrium single pulse observation of T2 (DESPOT2) method [16], T2 fast acquisition relaxation mapping (T2 FARM) methods [17–19], etc. However, due to the sensitivity to magnetic field inhomogeneity, DESPOT2 and T2 FARM methods cannot accurately measure the T2 values of tissues, while the stability of MESE method brings it to be the most suitable technique for T2 mapping [20, 21]. Regarding this method, two or more spin-echoes will need to be acquired in a single repetition time (TR) duration. The signal intensity (SI) of MESE sequence can be generally expressed as the following equation:

1 $$SI = K*N\left( H \right)*e^{{\left( { - \frac{TE}{{T2}}} \right)}} *\left[ {1 - e^{{\left( { - \frac{TR}{{T1}}} \right)}} } \right]$$

where SI is the measured signal intensity, *K* is constant, N(H) represents proton density, TR and echo time (TE) are known parameters. Therefore, T2 value can be calculated by mono-exponential fitting according to the above formula, and at least two echoes are needed theoretically. To improve the precision, more echoes are needed to be involved in the calculation. Based on MESE method, the T2 mapping sequence involved 9 echoes on 1.5 T MRI scanner and 8 echoes on 3.0 T MRI scanner in our study, and the additional acquisition time was 4′22″ and 5′15″ for 1.5 T and 3.0 T MR scanner respectively.

### Study subjects

This study was approved by the Institutional Ethics Committee of our hospital, and written informed consent was obtained from all subjects before the examination. A total of 54 healthy subjects and 139 patients with uterine lesions were enrolled in this study from September 2020 to December 2021. Pathological results of each uterine lesion were confirmed after surgical operations.

The inclusion criteria for healthy subjects were as follows: (1) childbearing-age healthy women; (2) no obvious lesions of the uterus and ovary through ultrasound examination; and (3) no contraindication for MRI examination. The exclusion criteria were as follows: (1) positive signs of uterus or ovary through MRI examination; (2) severe image artifacts due to intestinal peristalsis, breathing or body movement; and (3) the thickness of the junctional zone was too small (less than 3 mm) to measure. Among all healthy subjects, two subjects were excluded due to the appearance of myoma, while another two subjects were excluded due to severe image artifact and too thin junctional zone (thickness < 3 mm) respectively. Finally, 50 healthy subjects (age: 36.7 ± 5.9 years, age range: 21–48 years) containing 250 ROIs were included in the study (Fig. 1).

**Fig. 1:** Inclusion and exclusion flowchart for healthy subjects and patients

The inclusion criteria for patients were as follows: (1) patients with suspected uterine lesions recommended by clinical gynecologist (Weihong Lu with 8 years of gynecological experience), and (2) the lesion was found for the first time and did not receive any clinical treatment. The exclusion criteria were as follows: (1) severe image artifacts due to intestinal peristalsis, breathing or body movement; (2) the maximum diameter of the tumor was smaller than 5 mm; (3) myoma with necrosis; and (4) patients with uncertain pathology after operation. Among all patients, 4 patients with severe image artifacts, 2 patients with uncertain pathology, 1 patient with necrotic myoma, and 6 patients with tumors smaller than 5 mm were excluded. Finally, 126 patients (age: 46.2 ± 9.8 years, age range: 25–76 years) containing 133 lesion ROIs were included in the study (Fig. 1).

### Data acquisition

Healthy subjects underwent non-contrast routine uterus MRI examination with an additional T2 mapping sequence on a 1.5 T MRI scanner (Amira 1.5 T; Siemens Healthcare, Erlangen, Germany) first and then moved to the 3.0 T MRI scanner (Discovery MR750w; GE Healthcare, Milwaukee, WI, USA) to finish the corresponding T2 mapping data acquisition. For patients with uterine lesions, they finished the T2 mapping data acquisition on the above 1.5 T MRI first and then completed the routine contrast-enhanced uterus MRI examinations with an additional T2 mapping sequence on the above 3.0 T MRI scanner. The T2 mapping sequence was implemented before the contrast injection, and all examinations were finished on the same day for each participant. The 13-channel and 16-channel torso phased array coils with their corresponding integrated spine matrix coils were equipped as receivers on the 1.5 T and 3.0 T scanners, respectively.

To improve comfort for subjects during scanning, the foot-first supine position was used. The sequences and detailed acquisition parameters on the 1.5 T scanner were as follows: (1) axial T1-weighted imaging (T1WI); (2) T2-weighted imaging (T2WI); (3) fat-saturated T2WI; (4) diffusion-weighted imaging (DWI) with b-values of 0, 50, 800 s/mm2; (5) sagittal fat-saturated T2WI; (6) dynamic contrast enhancement using axial three-dimensional volumetric interpolated breath-hold examination (3D VIBE) sequences at 30 s, 60 s, and 150 s after gadolinium injection; (7) sagittal and coronal 3D VIBE sequences were also acquired at 90 s and 120 s to reveal the lesions. The routine sequences on the 3.0 T scanner were similar to those on the 1.5 T scanner. The detailed acquisition parameters for additional T2 mapping sequences based on the MESE method on these two scanners are listed in Table 1.

**Table 1:** The parameters of T2 Mapping sequences

	1.5 T	3.0 T
Repetition time (ms)	2000	1500
Echo time (ms)	(*n* = 9) 11.1/ 22.2/…/11.1*n	(*n* = 8) 9.05, 18.1 … 9.05*n
Slice thickness (mm) / gap (mm)	4.0 / 0.8	4.0 / 0.8
Field of view (mm^2^)	250 × 250	250 × 250
Acquisition matrix	256 × 192	288 × 192
Number of excitations	1.0	1.0
Acquisition time	4′22”	5′15”

### Image analysis

T2 maps were first calculated from T2 mapping images by monoexponential fitting using a custom code in MATLAB (R2017a; MathWorks, Natick, MA, USA). The T2 data of each participant were then transferred to Advantage Workstation 4.6 (AW4.6; GE Healthcare). Measurement was carried out on the workstation independently by two experienced radiologists (both of them had over 5 years of experience in cervical MRI), and the result was the mean value of two measurements.

Taking the axial T2WI images as a reference, the regions of interest (ROIs) were manually delineated on the maximum TE image of the T2 mapping sequence, which has best tissue contrast among all images with different TEs. For healthy subjects, ROIs were placed on the endometrium (size: ~ 40 mm^2^), junctional zone (size: ~ 100 mm^2^), external muscle layer (size: 200 mm^2^), gluteus maximus (size: 500 mm^2^), and subcutaneous fat (size: 500 mm^2^), and their T2 values can be obtained from T2 map. Take a 39-year-old healthy subject for example, Fig. 2(A) was the maximum TE image of T2 mapping sequence, on which each ROI was placed carefully (Fig. 2(B)), and Fig. 2(C) was the partial enlargement of Fig. 2(B). And then the T2 value of each ROI were measured from corresponding T2 map (Fig. 2(D)). For patients with uterine lesions, ROIs were placed on the maximum cross-section of the lesion (Fig. 2 (E–F) for example), and visible cystic necrosis was avoided during outlining. The ROIs from three consecutive layers were selected for signal averaging in each measurement. A total of 133 lesions were collected, including benign (adenomyosis: *n* = 21; myoma: *n* = 32; endometrial polyps: *n* = 28) and malignant lesions (cervical cancer: *n* = 23; endometrial carcinoma: *n* = 29).

**Fig. 2:** ROIs placement on image with maximum TE (99.9 ms, 1.5 T) of the T2 mapping sequence **A** from a 39-year-old healthy subject. **B** was the image with ROIs showed based on image **A**, and **C** was the partial enlargement of Fig. 2(B). On image (B), ROIs with label 1 to label 5 represented endometrium (area = 41mm^2^), junctional zone (area = 102mm^2^), external-myometrium (area = 201mm^2^), gluteus maximus (area = 500mm^2^) and subcutaneous fat (area = 500mm^2^) from inside to outside respectively, and their T2 values can be obtained from T2 map (**D**) directly. I and (**F**) were the image with maximum TE and the corresponding T2 map respectively from a 57-year-old endometrial carcinoma patient, and the ROI was placed carefully on the maximum cross-section of the lesion

### Statistics analysis

All statistical analyses were performed using SPSS software 25.0 (IBM Corp, Armonk, NY, USA). Data are expressed as the mean ± standard deviation. The intraclass correlation coefficient (ICC) was used to evaluate the interobserver consistency of the measured parameters. ICC values of less than 0.4, 0.41–0.75, and greater than 0.75 indicated poor, fair, and good agreement, respectively. The Kolmogorov‒Smirnov test was adopted to assess the normality of the data. The differences in T2 values in normal uterine structures and common benign and malignant tumors between different magnetic field strengths were compared by using the Wilcoxon match-pairs signed rank test. The differences in T2 values between common benign and malignant uterine lesions under the same magnetic field strength were also compared by using the Mann‒Whitney U test. The diagnostic efficacy was evaluated by ROC analysis, and AUC, sensitivity and specificity were obtained. The differences in AUCs were compared using the DeLong test.

## Results

### Clinical characteristics and interobserver reliability

After exclusion, a total of 50 healthy subjects and 126 patients were included in our study. The characteristics of the patients are listed in Table 2. The interobserver consistency of T2 values was good in all ROIs (all ICC > 0.85) (Table 3).

**Table 2:** The clinical characteristics for patients

Characteristics	
Number	126
Mean age (range)	46.2 ± 9.8 (25–76)
Pathology	
Adenomyosis	21
Myoma	32
Endometrial polyps	28
Cervical cancer	23 (Squamous cell carcinoma, 20; Adenocarcinoma, 3)
Endometrial carcinoma	29 (Endometrioid adenocarcinoma, 25; Mucinous adenocarcinoma, 2; Clear cell carcinoma, 2)

**Table 3:** Interobserver consistency of the T2 value

Groups	ICC (95% CI)	
	1.5 T MRI	3.0 T MRI
Healthy group		
Endometrium	0.96 (0.94–0.98)	0.97 (0.95–0.99)
Junctional zone	0.94 (0.89–0.96)	0.94 (0.90–0.97)
External-myometrium	0.91 (0.85–0.95)	0.88 (0.79–0.93)
Gluteus maximus	0.90 (0.84–0.94)	0.93 (0.88–0.96)
Subcutaneous fat	0.98 (0.96–0.99)	0.95 (0.91–0.97)
Patient group		
Adenomyosis	0.97 (0.93–0.99)	0.96 (0.91–0.98)
Myoma	0.94 (0.87–0.97)	0.94 (0.88–0.97)
Endometrial polyps	0.99 (0.98–1.00)	0.96 (0.91–0.98)
Cervical cancer	0.97 (0.94–0.99)	0.96 (0.90–0.98)
Endometrial carcinoma	0.94 (0.87–0.97)	0.92 (0.83–0.96)

*ICC* Intraclass correlation coefficient, *CI* Confidence interval

### Comparison of T2 values between 1.5 T and 3.0 T MRI in healthy subjects

In the healthy subject group, the mean T2 value in subcutaneous fat was the highest (134.8 ± 3.9 ms), followed by endometrium (110.9 ± 6.0 ms), external-myometrium layer (79.3 ± 5.4 ms), gluteus maximus (51.0 ± 4.4 ms), and junctional zone (50.0 ± 4.8 ms) under 1.5 T MRI. Similar results were found under 3.0 T MRI; the mean T2 value in subcutaneous fat was the highest (102.3 ± 3.2 ms), followed by endometrium (96.6 ± 3.5 ms), external-myometrium layer (75.7 ± 2.9 ms), gluteus maximus (44.3 ± 2.5 ms), and junctional zone (47.1 ± 2.5 ms). The T2 values in these tissues under 1.5 T MRI were significantly higher than those under 3.0 T MRI (all *p* < 0.05) (Figs. 3 and 4).

**Fig. 3:** The box & whiskers plot of T2 values in healthy group under 1.5 T and 3.0 T MRI (*: *p* < 0.05, **: *p* < 0.01)

**Fig. 4:** Pelvis axial T2 weighted image **A** and T2 maps under 1.5 T **B** and 3.0 T MRI **C** scanners from a 33-year-old healthy female. The T2 values of endometrium (pink arrow in (A)), junctional zone (orange arrow in (A)), external-myometrium layer (blue arrow in (A)), gluteus maximus (green arrow in (A)) and fat (yellow arrow in (A)) under 1.5 T scanner were 111.2 ms, 51.5 ms, 72.3 ms, 46.8 ms and 130.6 ms respectively. While T2 values for above structures under 3.0 T scanner were 102.8 ms, 47.2 ms, 64.7 ms, 43.7 ms and 101.5 ms respectively

### Comparison of T2 values between 1.5 T and 3.0 T MRI in patient group

In the patient group, the mean T2 value in endometrial carcinoma was the highest (104.4 ± 3.3 ms for 1.5 T; 95.8 ± 4.1 ms for 3.0 T), followed by cervical cancer (99.2 ± 4.1 ms for 1.5 T; 90.6 ± 6.2 ms for 3.0 T), endometrial polyps (96.9 ± 7.7 ms for 1.5 T; 85.9 ± 5.6 ms for 3.0 T), adenomyosis lesions (72.0 ± 4.2 ms for 1.5 T; 64.6 ± 4.1 ms for 3.0 T), and myoma (47.9 ± 4.6 ms for 1.5 T; 42.8 ± 3.1 ms for 3.0 T). The T2 values in these lesions under 1.5 T MRI were significantly higher than those under 3.0 T MRI (all *p* < 0.05) (Figs. 5 and 6).

**Fig. 5:** The box & whiskers plot of T2 values in patient group under both 1.5 T and 3.0 T MRI (**: *p* < 0.01)

**Fig. 6:** Typical T2 maps for benign and malignant lesions confirmed by pathology under 1.5 T and 3.0 T MRI. **A** axial T2WI image from a 51-year-old woman with subserous myoma of uterus (red arrow). **B** and (**C**) corresponding colored T2 maps under 1.5 T and 3.0 T MRI. The T2 values of this myoma under 1.5 T and 3.0 T MRI were 45.3 ms and 40.6 ms, respectively. The T2 values of adenomyosis (orange arrow) from a 44-year-old woman **D**–**F** were 73.5 ms and 68.3 ms under 1.5 T and 3.0 T MRI, respectively. **G**–**I** images belonged to a 65-year-old woman with cervical cancer (pink arrow), the T2 values of which were 95.1 ms and 90.2 ms under 1.5 T and 3.0 T MRI, respectively. **J**–**L** images were from a 61-year-old woman with endometrial carcinoma (dark red arrow), the T2 values of which were 108.5 ms and 99.7 ms under 1.5 T and 3.0 T MRI, respectively

### Comparison of T2 values between each two lesion-subgroup under a specific magnetic field

There were significant differences (*p* values < 0.05, Table 4) in T2 values between each two lesion-subgroup under 1.5 T or 3.0 T MRI except for the difference between endometrial polyps group and cervical cancer group.

**Table 4:** The T2 value comparisons between each two lesion-subgroup under 1.5 T and 3.0 T MRI respectively

Each two lesion-subgroup	*P* value	
	1.5 T MRI	3.0 T MRI
Adenomyosis vs. Myoma	< 0.001	< 0.001
Adenomyosis vs. Endometrial polyps	< 0.001	< 0.001
Adenomyosis vs. Cervical cancer	< 0.001	< 0.001
Adenomyosis vs. Endometrial carcinoma	< 0.001	< 0.001
Myoma vs. Endometrial polyps	< 0.001	< 0.001
Myoma vs. Cervical cancer	< 0.001	< 0.001
Myoma vs. Endometrial carcinoma	< 0.001	< 0.001
Endometrial polyps vs. Cervical cancer	0.173	0.100
Endometrial polyps vs. Endometrial carcinoma	< 0.001	< 0.001
Cervical cancer vs. Endometrial carcinoma	< 0.001	< 0.001

### Comparison of T2 values between benign and malignant lesions under a specific magnetic field

Uterine lesions of the patient group were divided into two subgroups, including the common benign group (adenomyosis, myoma and endometrial polyps) and common malignant group (cervical cancer and endometrial carcinoma). The mean T2 value of the benign group was significantly lower than that of the malignant group (*p* < 0.01) (Table 5 and Fig. 7) under 1.5 T MRI and 3.0 T MRI. The AUC of the T2 value under 1.5 T was 0.902, while it was 0.941 under 3.0 T in differentiating common benign and malignant lesions. The sensitivity, specificity and cutoff of the T2 value under 1.5 T MRI were 100%, 80.25% and 93.7 ms, respectively. The sensitivity, specificity and cutoff of the T2 value under 3.0 T MRI were 98.08%, 81.48% and 84.9 ms, respectively. The performance of the T2 value under 3.0 T MRI was significantly better than that under 1.5 T MRI (*p* = 0.02).

**Table 5:** The T2 value comparisons between benign and malignant lesions under 1.5 T and 3.0 T MRI

	1.5 T (ms)	3.0 T (ms)
Benign lesions (*n* = 81)	71.1 ± 22.0	63.4 ± 19.1
Malignant lesions (*n* = 52)	101.1 ± 4.5	93.5 ± 5.1
*P* value	< 0.001	< 0.001
AUC (95% CI)	0.90 (0.84–0.95)	0.94 (0.89–0.98)
Sensitivity	100%	98.08%
Specificity	80.25%	81.48%
Cutoff	93.7 ms	84.8 ms
Pairwise comparison of ROC curves	*p* = 0.02	

AUC Area under curve, *CI* Confidence interval, *ROC* Receiver operating characteristic

**Fig. 7:** The ROC curves of T2 value in differentiating common benign and malignant lesions under 1.5 T and 3.0 T MRI. The AUC of T2 value under 1.5 T was 0.902, while 0.941 under 3.0 T in differentiating common benign and malignant lesions

## Discussion

MRI diagnosis is not limited to imaging manifestations, and how to quantitatively evaluate the characteristics of lesions has become a hot research issue [22–25]. The transverse relaxation time (T2) of the tissue is similar to the longitudinal relaxation time (T1) and proton density (PD), all of which are intrinsic physical characteristics of the tissue in MRI. The T2 value can be used to assess tissue composition and reflect the water content of the tissue. The T2 value of a certain tissue was relatively constant under different conditions, which is of great significance for the study of lesions [26].

In our study, we found that the T2 values of normal tissues and uterine lesions at 3.0 T were lower than those at 1.5 T (Fig. 3 and Fig. 5), which was in line with the principle that the T2 value decreased in most tissues as field strength increased [27].

In the patient group, the T2 value of endometrial carcinoma was the highest, followed by cervical cancer, endometrial polyps, and adenomyotic lesions, while the T2 value of myoma was the lowest (Fig. 5). Endometrial carcinoma is a kind of epithelial malignant tumor originating from the endometrium, which is composed of glands similar to the normal endometrium. The glandular epithelium sprouted, proliferated and tangled in clusters [28]. Therefore, it was not difficult to explain why the T2 value of endometrial carcinoma (104.4 ± 3.3 ms at 1.5 T) was slightly lower than that of normal endometrium (110.9 ± 6.0 ms at 1.5 T). Cervical cancer is derived from immature cervical cells that experience abnormal proliferation and poor differentiation [29]. The T2 value of cervical cancer was 99.2 ± 4.1 ms at 1.5 T and 90.6 ± 6.2 ms at 3.0 T, which was consistent with results reported by Li et al. [30].

Endometrial polyps are aroused by focal excessive hyperplasia of the endometrium. They are composed of dense fibrous tissue, thick blood vessels and endometrial glands; thus, the T2 value of endometrial polyps was determined by these three structures. Due to the mixture of fibrous tissue, which contained less water, the T2 value of endometrial polyps (96.9 ± 7.7 ms at 1.5 T MRI) was lower than that of endometrial carcinoma and cervical cancer. Adenomyosis is caused by endometrial glands and stroma invading the myometrium, which was accompanied by old hemorrhage in general. Therefore, the T2 value of adenomyosis integrates the T2 value of the endometrial gland, stroma, myometrium and old hemorrhage. Due to the existence of stroma and hemorrhage, the T2 value of adenomyosis was lower than that of the normal external-myometrium layer (72.0 ± 4.2 ms vs. 79.3 ± 5.4 ms at 1.5 Myoma is s mainly formed by the proliferation of smooth muscle cells and fibrous connective tissue. In our study, the T2 value of the myoma was slightly lower than that of the gluteus maximus (47.9 ± 4.6 ms vs. 51.0 ± 4.4 ms at 1.5).

In our study, we also compared the T2 values between benign and malignant tumors preliminarily. The T2 values of benign tumors were significantly lower than those of malignant tumors, which can be explained by their different composition structures. Moreover, the ROC curve comparison of the T2 value in differentiating benign and malignant tumors between 1.5 T and 3.0 T MRI showed that the diagnostic performance of the T2 value under 3.0 T (AUC = 0.94) was significantly higher than that under 1.5 T MRI (AUC = 0.90).

This study had several limitations. First, the T2 value of the healthy group was only acquired from women of childbearing age. Therefore, the result of this part could only be the reference to this age group. Second, motion-related artifacts caused by respiration on T2 mapping images influenced the measurements T2 value, especially in 3.0 T MRI in a small number of patients, which were excluded from our study. It was better to consider using a motion-insensitive sequence or motion correction technique to improve the T2 mapping accuracy. Third, we all adopted recommended default acquisition parameters for T2 mapping sequences to ensure the image quality, thus the parameters under two field strengths were not identical, which might cause T2 fitting variance. Future study with exactly the same acquisition parameters under different field strengths should be made to further verify the results. Last, this study only considered cervical cancer and endometrial carcinoma as malignant tumors but did not involve other malignant tumors, such as uterine sarcoma, malignant hydatidiform mole or choriocarcinoma, due to the limited number of cases. And malignant tumors were not further classified according to pathological classification to verify the performance of T2 mapping. Although this preliminary study had the above limitations, the results build a foundation for further quantitative studies regarding uterine tumors.

## Conclusion

The T2 mapping technique provides an effective tool for quantifying normal uterine tissues, benign and malignant lesions. It can be applied to distinguish between benign and malignant lesions, especially under 3.0 T MRI, offering a new nonenhanced imaging tool for the further quantitative study of uterine tumors.

## Data Availability

The datasets used and/or analyzed during the current study are available from the corresponding author on reasonable request.

## Abbreviations

MRI: Magnetic resonance imaging
ROC: Receiver operating characteristic
AUC: Area under curve
MESE: Multi-echo spin-echo
DESPOT2: Driven equilibrium single pulse observation of T2
T2 FARM: T2 Fast acquisition relaxation mapping
TR: Repetition time
TE: Echo time
SI: Signal intensity
T1WI: T1-Weighted imaging
T2WI: T2-Weighted imaging
DWI: Diffusion-weighted imaging
3D VIBE: Three-dimensional volumetric interpolated breath-hold examination
ROI: Region of interest
ICC: Intraclass correlation coefficient

## References

[1] Siegel RL, Miller KD, Fuchs HE, Jemal A (2021). Cancer statistics, 2021. CA Cancer J Clin.

[2] Xia C, Dong X, Li H (2022). Cancer statistics in China and United States, 2022: profiles, trends, and determinants. Chin Med J (Engl).

[3] Testa AC, Di Legge A, De Blasis I (2014). Imaging techniques for the evaluation of cervical cancer. Best Pract Res Clin Obstet Gynaecol.

[4] Garcia-Reyes K, Passoni NM, Palmeri ML (2015). Detection of prostate cancer with multiparametric MRI (mpMRI): effect of dedicated reader education on accuracy and confidence of index and anterior cancer diagnosis. Abdom Imaging.

[5] Cheng HL, Stikov N, Ghuge NR (2012). Practical medical applications of quantitative MR relaxometry. J Magn Reson Imaging.

[6] Hepp T, Kalmbach L, Kolb M, Martirosian P, Hilbert T, Thaiss WM, Notohamiprodjo M, Bedke J, Nikolaou K, Stenzl A, Kruck S, Kaufmann S (2022). T2 mapping for the characterization of prostate lesions. World J Urol.

[7] Lee CH (2019). Quantitative T2-mapping using MRI for detection of prostate malignancy: a systematic review of the literature. Acta Radiol.

[8] Meng T, He N, He H (2020). The diagnostic performance of quantitative mapping in breast cancer patients: a preliminary study using synthetic MRI. Cancer Imaging.

[9] Kaggie JD, Deen S, Kessler DA (2019). Feasibility of quantitative magnetic resonance fingerprinting in ovarian tumors for T1 and T2 mapping in a PET/MR setting. IEEE Trans Radiat Plasma Med Sci.

[10] Ghosh A, Singh T, Bagga R (2018). T2 relaxometry mapping in demonstrating layered uterine architecture: parameter optimization and utility in endometrial carcinoma and adenomyosis: a feasibility study. Br J Radiol.

[11] Mittal S, Pradhan G, Singh S (2019). T1 and T2 mapping of articular cartilage and menisci in early osteoarthritis of the knee using 3-Tesla magnetic resonance imaging. Pol J Radiol.

[12] Bristela M, Skolka A, Eder J (2019). T2 mapping with 3.0 T MRI of the temporomandibular joint disc of patients with disc dislocation. Magn Reson Imaging.

[13] Tzimas G, Rotzinger DC, Muller O (2019). Myocardial oedema detected by T2-mapping: a key marker of recent ischaemia after resuscitated sudden cardiac death. Eur Heart J Cardiovasc Imaging.

[14] Arcari L, Camastra G, Ciolina F, Danti M, Cacciotti L (2022). T1 and T2 mapping in uremic cardiomyopathy: an update. Card Fail Rev.

[15] Wiggermann V, Vavasour IM, Kolind SH, MacKay AL, Helms G, Rauscher A (2020). Non-negative least squares computation for in vivo myelin mapping using simulated multi-echo spin-echo T2 decay data. NMR Biomed.

[16] Crooijmans HJ, Scheffler K, Bieri O (2011). Finite RF pulse correction on DESPOT2. Magn Reson Med.

[17] McKenzie CA, Chen Z, Drost DJ, Prato FS (1999). Fast acquisition of quantitative T2 maps. Magn Reson Med.

[18] Ben-Eliezer N, Sodickson DK, Shepherd T, Wiggins GC, Block KT (2016). Accelerated and motion-robust in vivo T2 mapping from radially undersampled data using bloch-simulation-based iterative reconstruction. Magn Reson Med.

[19] Fatemi Y, Danyali H, Helfroush MS, Amiri H (2020). Fast T2 mapping using multi-echo spin-echo MRI: a linear order approach. Magn Reson Med.

[20] Giri S, Chung Y-C, Merchant A (2009). T2 quantification for improved detection of myocardial edema. J Cardiovasc Magn Reson.

[21] Dvorak AV, Ljungberg E, Vavasour IM (2021). Comparison of multi echo T2 relaxation and steady state approaches for myelin imaging in the central nervous system. Sci Rep.

[22] Kvernby S, Flejmer AM, Dasu A, Bolger AF, Ebbers T, Engvall JE (2022). T1 and T2 mapping for early detection of treatment-related myocardial changes in breast cancer patients. J Magn Reson Imaging.

[23] Sathiadoss P, Schieda N, Haroon M (2022). Utility of quantitative T2-mapping compared to conventional and advanced diffusion weighted imaging techniques for multiparametric prostate MRI in Men with hip prosthesis. J Magn Reson Imaging.

[24] Kasar S, Ozturk M, Polat AV (2022). Quantitative T2 mapping of the sacroiliac joint cartilage at 3T in patients with axial spondyloarthropathies. Eur Radiol.

[25] Keerthivasan MB, Galons JP, Johnson K (2022). Abdominal T2-weighted imaging and T2 mapping using a variable flip angle radial turbo spin-echo technique. J Magn Reson Imaging.

[26] Cheng HL, Stikov N, Ghuger NR (2012). Practical medical applications of quantitative MR relaxometry. J Magn Resonan Imaging.

[27] Baeßler B, Schaarschmidt F, Stehning C, Schnackenburg B, Maintz D, Bunck AC (2015). A systematic evaluation of three different cardiac T2-mapping sequences at 1.5 and 3T in healthy volunteers. Eur J Radiol.

[28] Huvila J, Pors J, Thompson EF, Gilks CB (2021). Endometrial carcinoma: molecular subtypes, precursors and the role of pathology in early diagnosis. J Pathol.

[29] Johnson CA, James D, Marzan A, Armaos M (2019). Cervical cancer: an overview of pathophysiology and management. Semin Oncol Nurs.

[30] Li S, Zhang Z, Liu J (2021). The feasibility of a radial turbo-spin-echo T2 mapping for preoperative prediction of the histological grade and lymphovascular space invasion of cervical squamous cell carcinoma. Eur J Radiol.

